# Effect of parathyroid hormone on early chondrogenic differentiation from mesenchymal stem cells

**DOI:** 10.1186/s13018-014-0068-5

**Published:** 2014-08-01

**Authors:** Yun Zhang, Ken Kumagai, Tomoyuki Saito

**Affiliations:** 1 Department of Orthopaedic Surgery and Muscloskeletal Science, Graduate School of Medicine, Yokohama City University, 3-9 Fukuura, Kanazawa-ku 236-0004, Yokohama, Japan

**Keywords:** Parathyroid hormone, Chondrogenic differentiation, Mesenchymal stem cells

## Abstract

**Background:**

Treatment of articular cartilage injuries remains a difficult challenge due to the limited capacity for intrinsic repair. Mesenchymal stem cells (MSCs) can differentiate into chondrocytes under certain culture conditions. This study focused on the modulatory effects of parathyroid hormone (PTH) on chondrogenic differentiation from MSCs.

**Methods:**

MSCs were treated with various concentrations of PTH under chondrogenic pellet culture condition. RNA was isolated for real-time polymerase chain reaction (PCR) and gene expressions of collagen type II α1 chain (Col2a1), collagen type X α1 chain, collagen type I α1 chain, SRY-box9 (Sox9), and type 1 PTH/PTHrP receptor (PTH1R) were examined. Chondrogenic differentiation was also evaluated by histological findings.

**Results:**

PTH had opposite effects on chondrogenesis, depending on the concentration. A low to moderate concentration of PTH promoted chondrogenic differentiation of MSCs with increased expression of Sox9, Col2a1, and PTH1R, whereas chondrogenesis of MSCs was inhibited rather than stimulated with a higher concentration of PTH.

**Conclusion:**

This study provides insights into the modulatory effect of PTH on chondrogenic differentiation from MSCs and the therapeutic potential for cartilage regeneration. Based on clinical experience regarding the efficacy and safety of PTH for bone metabolism, PTH may also be useful clinically for cartilage repair.

## Background

Treatment of articular cartilage injuries remains a difficult challenge due to the limited capacity for intrinsic repair. Tissue engineering approaches have been introduced as treatment options for cartilage repair. Treatment efficacy depends entirely on the cells in the grafted site, particularly the small subset of stem and progenitor cells that are capable of generating new tissue [1]. Thus, cell-based approaches are key to successful tissue engineering [2].

Mesenchymal stem cells (MSCs) are the most commonly used cell source with a high self-renewal capacity, multilineage potential, and easy isolation from several human tissues including bone marrow [3],[4]. MSCs can differentiate into chondrocytes under certain culture conditions [5],[6] and have been used for cartilage regeneration medicine by many researchers [7],[8]. Therefore, a number of research efforts are directed to the isolation of progenitor cells and the understanding of the mechanisms involved in their chondrogenic differentiation.

Parathyroid hormone (PTH) is known as an 84-amino acid protein that regulates bone remodeling and calcium homeostasis. When PTH is administrated intermittently as a pharmacological agent, exogenous PTH has been shown to exert significant anabolic effects. Several studies indicated that PTH(1–34) also affects chondrocyte. PTH(1–34) inhibits the terminal differentiation of articular chondrocytes and the progression of osteoarthritis (OA) [9],[10]. In parallel with the suppression of chondrocyte hypertrophy, PTH(1–34) stimulates chondrocyte proliferation and differentiation in the early stage [11]–[15]. However, the effects of PTH on chondrogenic differentiation of MSCs remain to be elucidated. We hypothesized that PTH promotes early chondrogenic differentiation from MSCs. Here, we show the investigation of the modulatory effect of PTH on chondrogenic differentiation from MSCs.

## Materials and methods

### Culture of MSCs

Murine bone marrow-derived MSCs (Cyagen Biosciences, Santa Clara, CA, USA) were expanded in a monolayer culture with mesenchymal stem cell growth medium (GUXMX-90011, Cyagen Biosciences) supplemented with 10% fetal bovine serum, 100 units/mL penicillin, 100 μg/mL streptomycin, and glutamine at 37°C with 5% CO_2_ until the cells reached 80% confluence. The cells were then trypsinized and frozen in liquid nitrogen for later use. After thawing and monolayer expansion, cells at passage 5 or 6 were harvested and subjected to pellet formation and chondrogenic differentiation.

### Induction of chondrogenic differentiation and PTH administration

Pellets of 2.5 × 10^5^ MSCs were formed by centrifugation at 200 g for 5 min in 15-mL centrifuge tubes or 1.5-mL microcentrifuge tubes. After incubation at 37°C in 5% CO_2_ for 4 days, pellets were transferred to 96-well U-bottomed plates. Cells were exposed to chondrogenic medium (high-glucose DMEM with 0.1 μM dexamethasone, 0.17 mM ascorbic acid-2 phosphate, 5 μg/mL insulin, 5 μg/mL transferrin, 5 ng/ml selenous acid, 0.35 mM L-proline, 100 units/mL penicillin, and 100 μg/mL streptomycin) supplemented with 10 ng/mL transforming growth factor-β3 (TGF-β3). To detect the concentration dependency of PTH(1–34) treatment of TGF-β-driven chondrogenesis, TGF-β-enriched chondrogenic medium was supplemented with different concentrations of PTH (0.1, 1, 10, and 100 nM). The medium was changed every 2 or 3 days. Chondrogenic pellets were harvested at 3, 7, or 21 days.

### Histological analyses

After 3 weeks of culture, pellets were fixed overnight at 4°C in 4% paraformaldehyde solution, dehydrated with ethanol, washed with xylene, and embedded in paraffin. Sections at 5 μm thickness were cut from the paraffin blocks and mounted on glass slides. The sections were deparaffinized with xylene and ethanol prior to staining. To detect proteoglycan synthesis as an indicator of cartilage production, the sections were stained with Alcian Blue according to the standard protocol. For immunohistochemical staining of collagen type II, the sections were treated with 1 mg/ml hyaluronidase (Sigma, St. Louis, MO, USA) in PBS (pH 5.0) for 30 min at room temperature. After blocking nonspecific binding with 3% bovine serum albumin in PBS, rabbit anti-type II collagen antibody (Novus Biologicals, Littleton, CO, USA) was incubated overnight at 4°C. The next day, slides were washed in PBS and incubated with biotinylated anti-rabbit IgG antibody for 45 min at room temperature. Reaction was visualized by incubation with the avidin-biotin-peroxidase reagent included in the Vectastain ABC Kit (Vector Laboratories, Burlingame, CA, USA) followed by color development with 3-3′ diaminobenzidinetetrahydrochloride (Dojindo, Kumamoto, Japan). Finally, the sections were counterstained with hematoxylin and mounted with coverslips. Cartilage tissue from mouse knee joint was used for control staining of collagen type II. Normal rabbit IgG was used as an isotype control.

### Western blot analysis

For total protein extraction, pellets were homogenized and incubated with lysis buffer containing 20 mM Tris-HCl (pH 7.5), 150 mM NaCl, 1 mM Na_2_EDTA, 1 mM EGTA, 1% NP-40, 0.1% sodium dodecyl sulfate, 1 mM Na_3_VO_4_, and protease inhibitor cocktail (Nacalai tesque, Kyoto, Japan) for 30 min on ice and centrifuged at 15,000 rpm for 20 min at 4°C. Proteins were separated by 10% sodium dodecyl sulfate-polyacrylamide gel electrophoresis (SDS-PAGE) and transferred onto a polyvinylidene fluoride (PVDF) membrane. The membranes were incubated overnight at 4°C with rabbit primary antibodies against type 1 PTH/PTHrP receptor (PTH1R) (LifeSpan Biosciences, Seattle, WA, USA), SRY-box9 (Sox9) (Millipore, Temecula, CA, USA), Runt-related transcription factor 2 (Runx2) (Novus Biologicals, Littleton, CO, USA) and β-actin (Novus Biologicals). The membranes were washed and incubated with horseradish peroxidase labeled anti-rabbit IgG (Kirkegaard and Perry Laboratories, Gaithersburg, MD, USA) for 60 min at room temperature. After a washing step, bands were visualized by ECL Prime Western blotting detection reagent (GE Healthcare, Piscataway, NJ, USA) and analyzed using a luminescent image analyzer equipped with a cooled CCD camera (LAS 1000, Fujifilm, Tokyo, Japan).

### Total RNA isolation and RT-PCR

Total RNA was isolated from homogenized pellets using Trizol reagent (Invitrogen, Carlsbad, CA, USA). RNA was quantified by measuring absorbance at 260 nm, and the quality was assessed by determining the 260/280 nm absorbance ratio. First-strand cDNA synthesis was performed with 0.5 μg or 1 μg total RNA in a total volume of 20 μl using an iScript™ advanced cDNA synthesis kit (BIO-RAD, Richmond, CA, USA). Gene expressions of collagen type II α1 chain (Col2a1), collagen type X α1 chain (Col10a1), collagen type I α1 chain (Col1a1), Sox9, and PTH1R were examined with quantitative real-time PCR. The primers used in this study were listed in Table 1. Quantitative real-time PCR was carried out using SsoAdvanced™ SYBR Green supermix (BIO-RAD) on a CFX96™ real-time PCR detection system (BIO-RAD) in a 20-μl reaction volume. Expression of gene of interest was normalized to GAPDH expression.

**Table 1:** Primers used for real-time RT-PCR

**Gene**	**Direction**	**Sequences (5′–3′)**
Sox9	Forward	TACGACTGGACGCTGGTGCC
Sox9	Reverse	CCGTTCTTCACCGACTTCCTCC
Col2a1	Forward	CTGACCTGACCTGATGATACC
Col2a1	Reverse	CACCAGATAGTTCCTGTCTCC
Col10a1	Forward	CGAGGTATGCTTGATCTG
Col10a1	Reverse	GACAGTCCAGTTCTTCAT
Col1a1	Forward	TGACTGGAAGAGCGGAGAGT
Col1a1	Reverse	TCTCTCCAAACCAGACGTGC
PTH1R	Forward	CTCCTTCTCTGCTGCCCAGT
PTH1R	Reverse	TGCTGTGTGCAGAACTTCCT
GAPDH	Forward	TGAAGCAGGCATCTGAGGG
GAPDH	Reverse	CGAAGGTGGAAGAGTGGGAG

### Statistical analysis

All experiments were repeated at least three independent times. All data are presented as the mean ± SEM. The analysis was done using SigmaStat 3.5 software (Systat Software Inc., Richmond, CA, USA). The nonparametric Kruskal-Wallis test was used to test for significant differences among the test groups. When a significant difference was detected, Steel's *post hoc* test was performed to compare each of the treatments with a control. An adjusted *P* value < 0.05 was considered statistically significant.

## Results

### Histological findings

Chondrogenic differentiation was confirmed with Alcian Blue staining for proteoglycan synthesis. Positive staining with Alcian Blue was identified in all treatment groups (Figure 1A,B,C,D,E). Among the groups, stronger staining was observed with 1 and 10 nM PTH, whereas less intense staining was seen with 100 nM PTH. Regarding cellular morphology, sections from cells treated with 10 nM PTH exhibited more chondrocyte-like cells with large round nuclei than cells treated with 100 nM PTH. To further address chondrogenic differentiation, we examined the deposition of type II collagen, which is a major component of the cartilage extracellular matrix (Figure 1F,G,H,I,J). Expression of type II collagen was partially localized in 0 nM PTH control. Improved expression was found in 10 nM PTH. In contrast, almost negative expression was shown in 100 nM PTH.

**Figure 1:** **Histological findings of chondrogenic pellet cultures of MSCs treated with PTH for 21 days.** Upper panels **(A–E)** show Alcian Blue staining, and lower panels **(F–J)** show immunohistochemical staining of collagen type II. PTH was administrated at various doses: 0 **(A, F)**, 0.1 **(B, G)**, 1 **(C, H)**, 10 **(D, I)**, or 100 nM **(E, J)**. Immunohistochemical staining of mouse cartilage tissue using anti-collagen type II antibody **(K)** and normal rabbit IgG (**L**, as a negative control). Note that no background staining is observed in the section incubated with normal rabbit IgG. Scale bars = 100 μm.

### Effect of PTH on protein expression in chondrogenic differentiation

Protein expressions of PTH1R, Sox9, and Runx2 were detected by Western blotting (Figure 2). Positive expression of PTH receptor was confirmed in 0 − 10 nM PTH, whereas the intensity was remarkably reduced in 100 nM PTH. Protein expression of Sox9, a master regulator of chondrogenesis, was identified 3 weeks after chondrogenic differentiation from MSCs. Strong bands were present in 1 and 10 nM PTH and less intense one in 100 nM. Runx2, a transcription factor that promotes chondrocyte hypertrophy, was not intensely expressed in any PTH concentration.

**Figure 2:** **Effect of PTH on protein expression in chondrogenic pellet culture for 21 days.** Expression of PTH1R, Sox9, and Runx2 in various concentrations of PTH was analyzed using Western blotting.

### Effect of PTH on collagen expression in early stage of chondrogenic differentiation

To determine whether PTH modulates the early stage of chondrogenic differentiation of MSCs, gene expression of type II collagen as a marker of chondrogenesis was analyzed when cells were treated with various doses of PTH (Figure 3A). Relative mRNA expression of Col2a1 was significantly reduced with 100 nM PTH at days 3, 7, and 21 (*P* < 0.05, vs. 0 nM PTH). In contrast, treatment with 1 and 10 nM PTH resulted in significantly increased expression of Col2a1 at days 7 and 21 (*P* < 0.05, vs. 0 nM PTH). To assess the phenotypic change of hypertrophy during chondrogenesis of MSCs, gene expression of type X collagen as a marker of chondrogenic hypertrophy was also examined (Figure 3B). Relative mRNA expression of Col10a1 was not significantly changed with different doses of PTH at days 3, 7, and 21. To further characterize the effect of PTH on chondrogenic differentiation of MSCs, gene expression of type I collagen as a marker of hypertrophic or osteogenic differentiation was investigated (Figure 3C). We observed no significant difference in relative mRNA expression levels of Col1a1 at days 3, 7, and 21 among the various dose groups.

**Figure 3:** **Effect of PTH on collagen expression in chondrogenic pellet culture for 3, 7, and 21 days.** Relative mRNA levels of Col2a1 **(A)**, Col10a1 **(B)**, and Col1a1 **(C)** following PTH treatment are compared with expression in the control (0 nM PTH) (*n* = 8 for each dose). *P < 0.05 vs. control group (Steel's test).

### Effect of PTH on activation of Sox9 and PTH receptor during chondrogenic differentiation of MSCs

To assess the effect of PTH on the key transcription factor involved in chondrogenic differentiation, gene expression of Sox9 was analyzed (Figure 4A). Relative mRNA expression of Sox9 was significantly diminished in the presence of 100 nM PTH after days 3 and 21 (*P* < 0.05, vs. 0 nM PTH). In contrast, significantly increased levels of Sox9 were seen with 0.1 nM PTH at day 7, and 1 and 10 nM PTH at days 7 and 21 (*P* < 0.05, vs. 0 nM PTH). These expression patterns of Sox9 among the various doses were similar to those of Col2a1. To determine if the receptor is upregulated in response to PTH administration, gene expression of the PTH receptor was examined (Figure 4B). Relative mRNA expression of PTH1R was significantly decreased with 100 nM PTH at days 3, 7, and 21 (*P* < 0.05, vs. 0 nM PTH). In contrast, PTH1R was significantly increased with 1 and 10 nM PTH at days 7 and 21 (*P* < 0.05, vs. 0 nM PTH). The expression patterns for PTH1R were very similar to those for Sox9 and Col2a1.

**Figure 4:** **Effect of PTH on transcription factor involved in chondrogenic differentiation and response of PTH receptor.** In chondrogenic pellet culture for 3, 7, and 21 days. Relative mRNA levels of Sox9 **(A)** and PTH1R **(B)** following PTH treatment are compared with expression in the control (0 nM PTH) (*n* = 8 for each dose). *P < 0.05 vs. control group (Steel's test).

## Discussion

The present study demonstrated that chondrogenic differentiation of MSCs was modulated by PTH. The results revealed that PTH has opposite effects on chondrogenesis when administered at different concentrations. Namely, low to moderate concentrations of PTH promoted chondrogenic differentiation of MSCs, whereas chondrogenesis of MSCs was inhibited and not stimulated by a higher concentration of PTH.

This study was intended to test the hypothesis that PTH has a stimulatory effect on chondrogenic differentiation. An effect on induction of chondrogenesis with increased collagen type II was previously confirmed using a single concentration of PTH in growth plate chondrocytes [13] and MSCs from osteoarthritis patients [15]. In contrast, the inhibitory function of PTH on chondrocyte hypertrophy has been shown with reduced expression of collagen type X under conditions that promote chondrogenic differentiation [15],[16]. The constitutive expression of the PTH/PTHrP receptor in a bone morphogenetic protein-dependent differentiation system leads to a marked stimulation of chondrogenic and osteogenic development, whereas permanent application of the ligand PTH(1–34) results in opposite responses by stimulating the early and suppressing the late stages of osteo-/chondrogenic development [17]. These contrasting effects of PTH(1–34) on osteogenic and chondrocytic development seem to depend on the cellular state of differentiation. Our results were partially consistent with those previous reports. However, different from previous reports, we observed that expression of both Col2a1 and PTH1R was suppressed by a higher concentration of PTH. To our knowledge, no supportive studies have been published showing that the response to PTH during chondrogenic differentiation is opposite depending on a lower or higher concentration. Therefore, the modulatory effect of PTH on chondrogenic differentiation is likely to remain controversial.

PTH and PTHrP show homology in the amino-terminal (1–34) peptide fragments with high-affinity binding to PTH1R. Biological responses elicited by either ligand through this common PTH1R are largely indistinguishable, at least with regard to mineral ion homeostasis [18]. According to Weiss and colleagues [19], adding 0.1 ng/mL of PTHrP beginning on day 21 could suppress collagen type X deposition without any negative effects on chondrogenic differentiation, whereas higher concentrations (10 or 100 ng/mL) or earlier treatment (from day 0) would lead to the suppression of chondrogenesis. These contradictory effects of PTHrP on chondrogenic differentiation seem to be applicable to PTH on the basis of high similarity in the biological function [20]. Physicians may be interested in PTH rather than PTHrP because the former is currently available for clinical application. Therefore, several issues regarding the efficacy of PTH administration for successful cartilage repair need to be investigated further, including optimization of the concentration, treatment timing, and delivery method. The advantage of this study is that the investigations included a concentration-response range and examination of changes in expression of the exact genes.

The transcription factor Sox9 has been demonstrated to be a master regulator of the differentiation of mesenchymal cells into chondrocytes [21],[22]. The TGF-β signal plays an essential role to induce primary chondrogenesis [4],[23], which is mediated by up-regulation of Sox9 [24]. Furthermore, Sox9 is a target of PTH/PTHrP receptor signaling to maintain the chondrocyte phenotype and inhibit their maturation to hypertrophic chondrocytes in the growth plate [25]. Our results support the idea of a PTH/PTHrP receptor signal-dependent increase in Sox9 expression during chondrogenic differentiation from MSCs.

This study has several limitations including the concentration and timing for administration of PTH. Physiological PTH concentrations are much lower than those used in this study. However, in a number of in vitro studies examining the efficacy of PTH, the concentration tested is usually out of therapeutic ranges [9],[12],[13],[15],[16]. The response to PTH administration increases in a concentration-dependent manner, and the minimum effective concentration is higher than physiological levels [13],[26]. Therefore, we have chosen concentrations that significantly altered the cellular response and that showed the expected efficacy. The ability to reflect clinical relevance with cell culture models is difficult due to the lack of physiological conditions once cells are isolated from tissues and organs. The question is whether the output response is supportive of our understanding of the biology that will lead to decisions regarding translation of appropriate concentrations for assessment in human clinical testing. Furthermore, the relationship between the timing of exposure and the efficacy is unclear because PTH was continuously administered throughout the experimental period. For clinical use, PTH is intermittently administered when utilized for bone anabolic effects. Whether intermittent administration rather than continuous administration is effective for cartilage induction remains to be determined. This point is especially important for direct administration for therapeutic use. Further studies are required to extrapolate the translatable efficacy and safety in humans. For current therapeutic application, indirect treatment of human organ systems *ex vivo*, such as treatment prior to cell implantation, seems rational.

## Conclusions

This study provides insight into the modulatory effect of PTH on chondrogenic differentiation from MSCs. Ideal repair of injured cartilage involves replacement with hyaline cartilage and prevention of osteoarthritic changes. Several animal studies have shown that PTH has therapeutic potential for cartilage regeneration and protection as well as inhibition of progression of osteoarthritis [9],[10],[14]. PTH(1–34) has a stimulatory effect on bone formation with intermittent administration and is currently used as an anabolic drug for treatment of osteoporosis. Based on clinical experience with the efficacy and safety of PTH for bone metabolism, PTH may also be clinically useful for cartilage repair.

## Competing interests

The authors declare that they have no competing interests.

## Authors’ contributions

YZ, KK, and TS conceived and developed the study design. YZ and KK performed data acquisition and analysis. YZ and KK drafted the manuscript. All authors read and approved the final manuscript.

## References

[B1] MuschlerGFMiduraRJConnective tissue progenitors: practical concepts for clinical applicationsClin Orthop Relat Res2002395668010.1097/00003086-200202000-0000811937867

[B2] MuschlerGFNakamotoCGriffithLGEngineering principles of clinical cell-based tissue engineeringJ Bone Joint Surg Am200486-A154115581525210810.2106/00004623-200407000-00029

[B3] CaplanAIMesenchymal stem cellsJ Orthop Res1991964165010.1002/jor.11000905041870029

[B4] PittengerMFMackayAMBeckSCJaiswalRKDouglasRMoscaJDMoormanMASimonettiDWCraigSMarshakDRMultilineage potential of adult human mesenchymal stem cellsScience199928414314710.1126/science.284.5411.14310102814

[B5] JohnstoneBHeringTMCaplanAIGoldbergVMYooJUIn vitro chondrogenesis of bone marrow-derived mesenchymal progenitor cellsExp Cell Res199823826527210.1006/excr.1997.38589457080

[B6] SekiyaILarsonBLVuoristoJTRegerRLProckopDJComparison of effect of BMP-2, −4, and −6 on in vitro cartilage formation of human adult stem cells from bone marrow stromaCell Tissue Res200532026927610.1007/s00441-004-1075-315778851

[B7] RichardsonSMHoylandJAMobasheriRCsakiCShakibaeiMMobasheriAMesenchymal stem cells in regenerative medicine: opportunities and challenges for articular cartilage and intervertebral disc tissue engineeringJ Cell Physiol2010222233210.1002/jcp.2191519725073

[B8] WakitaniSImotoKYamamotoTSaitoMMurataNYonedaMHuman autologous culture expanded bone marrow mesenchymal cell transplantation for repair of cartilage defects in osteoarthritic kneesOsteoarthritis Cartilage20021019920610.1053/joca.2001.050411869080

[B9] ChangJKChangLHHungSHWuSCLeeHYLinYSChenCHFuYCWangGJHoMLParathyroid hormone 1–34 inhibits terminal differentiation of human articular chondrocytes and osteoarthritis progression in ratsArthritis Rheum2009603049306010.1002/art.2484319790062

[B10] SampsonERHiltonMJTianYChenDSchwarzEMMooneyRABukataSVO'KeefeRJAwadHPuzasJERosierRNZuscikMJTeriparatide as a chondroregenerative therapy for injury-induced osteoarthritisSci Transl Med20113101ra19310.1126/scitranslmed.3002214PMC320827121937758

[B11] HarringtonEKCoonDJKernMFSvobodaKKPTH stimulated growth and decreased Col-X deposition are phosphotidylinositol-3,4,5 triphosphate kinase and mitogen activating protein kinase dependent in avian sternaAnat Rec (Hoboken)201029322523410.1002/ar.2107219957341

[B12] HarringtonEKRoddyGWWestRSvobodaKKParathyroid hormone/parathyroid hormone-related peptide modulates growth of avian sternal cartilage via chondrocytic proliferationAnat Rec (Hoboken)200729015516710.1002/ar.2041617441208

[B13] IshikawaYWuLNGengeBRMwaleFWuthierREEffects of calcitonin and parathyroid hormone on calcification of primary cultures of chicken growth plate chondrocytesJ Bone Miner Res19971235636610.1359/jbmr.1997.12.3.3569076578

[B14] KudoSMizutaHTakagiKHirakiYCartilaginous repair of full-thickness articular cartilage defects is induced by the intermittent activation of PTH/PTHrP signalingOsteoarthritis Cartilage20111988689410.1016/j.joca.2011.04.00721571083

[B15] MwaleFYaoGOuelletJAPetitAAntoniouJEffect of parathyroid hormone on type X and type II collagen expression in mesenchymal stem cells from osteoarthritic patientsTissue Eng Part A2010163449345510.1089/ten.tea.2010.009120569194

[B16] ZeregaBCermelliSBiancoPCanceddaRCanceddaFDParathyroid hormone [PTH(1–34)] and parathyroid hormone-related protein [PTHrP(1–34)] promote reversion of hypertrophic chondrocytes to a prehypertrophic proliferating phenotype and prevent terminal differentiation of osteoblast-like cellsJ Bone Miner Res1999141281128910.1359/jbmr.1999.14.8.128110457260

[B17] HollnagelAAhrensMGrossGParathyroid hormone enhances early and suppresses late stages of osteogenic and chondrogenic development in a BMP-dependent mesenchymal differentiation system (C3H10T1/2)J Bone Miner Res1997121993200410.1359/jbmr.1997.12.12.19939421232

[B18] MannstadtMJuppnerHGardellaTJReceptors for PTH and PTHrP: their biological importance and functional propertiesAm J Physiol1999277F665F6751056422910.1152/ajprenal.1999.277.5.F665

[B19] WeissSHennigTBockRSteckERichterWImpact of growth factors and PTHrP on early and late chondrogenic differentiation of human mesenchymal stem cellsJ Cell Physiol201022384932004985210.1002/jcp.22013

[B20] ZhangWChenJZhangSOuyangHWInhibitory function of parathyroid hormone-related protein on chondrocyte hypertrophy: the implication for articular cartilage repairArthritis Res Ther20121422110.1186/ar389622971952PMC3580589

[B21] AkiyamaHChaboissierMCMartinJFSchedlAde CrombruggheBThe transcription factor Sox9 has essential roles in successive steps of the chondrocyte differentiation pathway and is required for expression of Sox5 and Sox6Genes Dev2002162813282810.1101/gad.101780212414734PMC187468

[B22] BiWDengJMZhangZBehringerRRde CrombruggheBSox9 is required for cartilage formationNat Genet199922858910.1038/879210319868

[B23] HengBCCaoTLeeEHDirecting stem cell differentiation into the chondrogenic lineage in vitroStem Cells2004221152116710.1634/stemcells.2004-006215579636

[B24] FurumatsuTTsudaMTaniguchiNTajimaYAsaharaHSmad3 induces chondrogenesis through the activation of SOX9 via CREB-binding protein/p300 recruitmentJ Biol Chem20052808343835010.1074/jbc.M41391320015623506

[B25] HuangWChungUIKronenbergHMde CrombruggheBThe chondrogenic transcription factor Sox9 is a target of signaling by the parathyroid hormone-related peptide in the growth plate of endochondral bonesProc Natl Acad Sci U S A20019816016510.1073/pnas.98.1.16011120880PMC14561

[B26] RickardDJWangFLRodriguez-RojasAMWuZTriceWJHoffmanSJVottaBStroupGBKumarSNuttallMEIntermittent treatment with parathyroid hormone (PTH) as well as a non-peptide small molecule agonist of the PTH1 receptor inhibits adipocyte differentiation in human bone marrow stromal cellsBone2006391361137210.1016/j.bone.2006.06.01016904389

